# Antioxidant and Teratogenic Activities of Formulated Agar Extracted from Brown Seaweed *Turbinaria conoides* against Zebrafish Larvae

**DOI:** 10.1155/2022/3520336

**Published:** 2022-07-11

**Authors:** Thabitha Aavula, Vignesh Narasimman, Saravanan Ramachandran, Radajurai Murugan, Murugavel Ponnusamy, Gururaja Perumal Pazhani, Sivaleela G

**Affiliations:** ^1^Native Medicine and Marine Pharmacology Laboratory, Department of Medical Biotechnology, Faculty of Allied Health Sciences, Chettinad Academy of Research and Education, Kelambakkam 603 103, Tamil Nadu, India; ^2^Department of Food Technology, M S Ramaiah University of Applied Sciences, Bangaluru, Karnataka, India; ^3^Center for Developmental Cardiology, Qingdao University, Qingdao 266021, China; ^4^SRM College of Pharmacy, SRM Institute of Science and Technology, Kattankulathur 603203, Tamil Nadu, India; ^5^Marine Biology Reginal Centre, Zoological Survey of India, Chennai 600 028, Tamil Nadu, India

## Abstract

This study examines the antioxidant and teratogenic effects of two different type's methods of formulating agar from *Turbinaria conoides* (*T. conoides*) using a zebrafish model. The agar was extracted using the aqueous extraction method and developed in two different formulations using separate procedures. Formulated agar1 (FA1) used a higher concentration of the ingredients while formulated agar 2 (FA2) had a lesser concentration. The two unique formulated agars (FAs) were studied using biochemical composition, Fourier infrared (FT-IR) spectroscopy, gas chromatography-mass spectroscopy (GC-MS), and scanning electron microscopy (SEM). The antioxidant activities of both FAs in vitro were shown to be significantly different (*P* < 0.05) at various concentrations (60–180 *μ*l/ml) in the study. The toxicity of the FAs was dose-dependent, with FA1 having the least teratogenic activity when compared to FA2. In comparison to FA2, FA1 was found to have higher antioxidant activity. At various concentrations (0.5, 0.25, and 0.125 *μ*g/ml), the teratogenic activity of two FAs was examined in zebrafish embryos (ZFE) at 24, 48, 72, and 96 hours post fertilization (hpf). Both FAs exhibit dose-dependent toxicity and increased antioxidant activity, and this can be utilized as an alternative for standard antioxidants, according to this study.

## 1. Introduction

Seaweeds/marine algae are a major part of the structurally diverse marine flora with several properties like antibacterial, anti-inflammatory, antiaging and anticarcinogenic. Seaweeds are rich in antioxidants and have potentially higher cosmetic effects due to the presence of several active ingredients. Cosmetic products derived from seaweed are increasingly preferred over synthetic compounds, with no harmful chemical compounds [1, 2]. Polysaccharides extracted from seaweeds play a pivotal role as humectants and moisturizers in cosmetic formulations, and can also be used as thickeners, gelling agents, film formers and emulsifiers [3]. *Turbinaria conoides* (*T. conoides*), brown algae which belong to the Sargassaceace family and the Fucales order, are a rich source of polysaccharides. The ethyl acetate extract of *Turbinaria conoides* was reported to have several properties like antibacterial, anticancer and higher antioxidant activity. Antioxidants are vital to reduce oxidative stress by removing the excess free radicals which have been associated with the emergence of degenerative processes in molecular biology, which encourage oxidative activities that are harmful to the body. The capacity of antioxidant chemicals in plants (carotenoids, polyphenols, polysaccharides, unsaturated fatty acids, vitamins, enzymes, and cofactors) to trap free radicals has inspired interest in employing them in preventative and curative phytotherapy [4]. *T. conoides* are a rich source of several phytochemical components such as sulphated polysaccharides, glucuronic acid, and alginic acid, and also contain compounds such as digestible proteins, mineral salts (K, Ca, and Fe), and polyunsaturated fatty acids [5]. Our laboratory had previously investigated the anti-skin cancer and antioxidant effects of FA from the brown seaweed *Laminaria digitata* [6], but this finding has not been reported using the standard FA method. Drug screening with zebrafish has several advantages, like increased efficiency, lower operating costs, shorter testing periods, easily controllable experimental conditions, and most significantly, increased genetic similarities between zebrafish and humans (approximately 70%) which makes the zebrafish a successful animal model [7]. Hence, the current study compared the antioxidant capabilities and toxicity of FA in zebrafish embryos (ZFEs).

## 2. Materials and Methods

### 2.1. Seaweed Collection

The brown seaweeds (*T. conoides*) were collected from the Gulf of Mannar (9.1278°N, 79.4662°E), Tamil Nadu, India, during the period of December 2020–January 2021. The brown seaweeds were known and confirmed by the Central Marine Fisheries Research Institute (CMFRI). Brown seaweeds were collected and then washed in fresh water to remove any undesired elements, such as other seaweed species. These samples were meticulously cleaned with seawater before being rinsed in double-distilled water. The seaweeds were dried in the shade and finely powdered with a blender before being stored at −20°C for subsequent investigation.

### 2.2. Extraction of Agar

To extract water-soluble polysaccharides, 20 g fine powdered seaweed samples were combined with 200 ml Milli-Q water and autoclaved at 121°C for 1 h. To remove seaweed debris, the extract was then filtered through Whatman No. 1 filter paper and centrifuged at 4500 rpm for 20 min. To produce a gel, the extract was maintained at room temperature [8].

### 2.3. Preparation of FAs

Agar processing methods have been developed in several countries, as illustrated in Figure 1, the extracted agar was transformed into a formulation using two distinct processes [9, 10].

### 2.4. Characterization of FAs

The colour, odour, consistency, sterility, and homogeneity were all employed to identify the characteristics of both FAs [11–13]. pH, vibrational testing, centrifugation tests, and physicochemical properties were all looked into [14, 15]. The information presented here pertains to three different determinations.

### 2.5. Biochemical Composition of FAs by Flame Emission Atomic (FEA) Spectroscopy

0.2 g of two FAs were mixed with HClO₄ and left undisturbed for 5 min. 5 ml of conc. HNO_3_ was mixed and incubated for 5 min followed by adding 5 ml of conc. HCl. The mixture was allowed to evaporate. An FEA spectrophotometer was used to analyze the filtrate. The minerals analyzed were calcium and phosphorus. The results were expressed as ppm and percentage [16].

### 2.6. Structural Characterization

#### 2.6.1. Fourier Transform Infrared Spectroscopy (FT-IR) of FAs

FT-IR qualitative analysis of two FAs was performed by using a Bruker Alpha instrument (USA) with the spectrum recorded between 4000 to 400 cm^−1^ [17].

#### 2.6.2. Gas Chromatography-Mass Spectrometry (GC-MS) of FAs

The GC-MS spectroscopic analysis was carried out (Agilent, Santa Clara, CA, USA). The detection of an electron ionization system with an activity force of 70 eV and a mass range of 30 to 650 m/*z* was utilized [18].

#### 2.6.3. Scanning Electron Microscope (SEM) of FAs

The structural characteristic of both FAs were designed with a JSM-5600 LV, SEM, (Jeol, Tokyo, Japan). The samples were analyzed at increasing temperatures (200°C, 400°C, 600°C, and 1200°C) with magnifications of 5.00 KX, 2.50 KX, 2.52 KX, and 1.00 KX [19].

### 2.7. In Vitro Antioxidant Assay

#### 2.7.1. (1,1,Diphenyl-2,picrylhydrazyl) DPPH Scavenging Activity

The DPPH radical scavenging assay was performed in increasing sample concentration of 50 *μ*l-100 *μ*g/ml. 200 *μ*l of methanolic DPPH solution was added and mixed thoroughly using a vortex mixer. The absorbance was measured at 517 nm in UV spectroscopy and the state was measured by using the following formula [20]:

(1) $$\begin{array}{c} DPPH\text{ scavenging assay}\left(\%\right)=\left[\left(A\;control-A\;sample\right)/A\;control\right]x100, \end{array}$$

where A control = absorbance of the control sample; A sample = absorbance of FA.

#### 2.7.2. H_2_O_2_ Radical Scavenging Activity

0.5 ml of FA solutions was added with 600 *μ*l H_2_O_2_ solution (40 Mm) to determine the H_2_O_2_ radical scavenging activity. The absorbance was then calculated at 230 nm in UV spectroscopy [16].

H_2_O_2_ scavenging activity (%) = [(A control−A sample)/A control] x 100,where A control = absorbance of the control sample; A sample = absorbance of FA.

#### 2.7.3. Total Antioxidant Activity (TAA)

The TAA of FAs was determined by using a total antioxidant capacity (TAC) solvent (0.6 M sulfuric acid, 28 mM sodium phosphate, and 4 mM ammonium molybdate). 0.2 ml FAs were mixed with 3 ml of the TAC reagent solution and then incubated in a water bath for 90 min. The readings of the reaction were then measured at 695 nm by using a UV-visible spectrophotometer [4].

(2) $$\begin{array}{c} TAA\left(\%\right)=\left[\left(A\;control-A\;sample\right)/A\;control\right]x100, \end{array}$$

where A control = absorbance of the control sample and A sample = absorbance of FA.

#### 2.7.4. 2,2-Azino-is-3-ethylbenzothiazoline-6-sulfonic Acid (ABTS) Activity

The ABTS solution absorbance was checked using 1 ml ABTS solvent with 60 ml methanol to attain the readings of 0.73 at 734 nm. The ABTS activity of FAs was compared with standard vitamin *E* at 734 nm in a UV-visible spectrophotometer [20].

(3) $$\begin{array}{c} ABTS\left(\%\right)=\left[\left(A\;control-A\;sample\right)/A\;control\right]x100, \end{array}$$

where A control = absorbance of the control sample and A sample = absorbance of FA.

### 2.8. Zebrafish Husbandry

At a temperature of 28°C, adult wild zebrafish were kept in dark and light for 10 to 14 hrs at a time. Natural spawning was used to gather viable eggs, which were then washed in distilled water the next morning. The E3 medium (34.8 g NaCl, 1.6 g KCl, 5.8 g CaCl_2_·2H_2_O, 9.78 g MgCl_2_·6H_2_O) was used to harvest and store embryos. For the teratogenic FAs investigation, coagulated and damaged eggs were removed and viable eggs were chosen [21].

### 2.9. Teratogenic Activities of FAs

At varied diluted concentrations (0.5, 0.25, and 0.125 *μ*g/ml), the teratogenic activity of the two distinct FAs was tested. A stereomicroscope was used to investigate the ZEF at various phases of growth [22].

### 2.10. Statistical Analysis

Each test was carried out in a triplicate manner, with the findings reported as the mean SD. Significance was defined as a *P* value of <0.05. IBM SPSS Statistics for Windows, version 22, was used for statistical analysis (IBM Corp., Armonk, N.Y., USA).

## 3. Results and Discussion

The wet weights of FAs obtained by FA1 84.2% and FA2 80.6% are mentioned in (Table 1). The chemicals and quantity have an impact on the yield and rate of an FA. Marine pharmacologist creates methods in the manufacturing business that maximize the yield and production rate of FA. They also want to cut waste and energy expenses at every step of the experiment [23]. The agar formulation methods and yield used for developing antioxidant properties for both the FAs from brown seaweed have been successful (*T. conoides*). The macroelements of FA1 were found to be high in Na (3.3%) when compared to FA2 being low in Na (2.23%). The macro elements of FA1 were found to be high in sodium Na (2.6 ± 0.3) compared to FA2 being low in Na (2.4 ± 0.2). The microelements in FA1 contained more copper (76.01 ± 0.4) than in FA2 (73.2 ± 0.5). The FA1 has higher sulphate content (39.78%) than the FA2 (37.25%), as shown in (Table 1).

Marine algae are rich sources of macroelements such as K, Ca, Na, and Mg. The results of FA were similar to *Sargassum wightii*, which also showed higher Na ions concentration. In *L. digitata,* higher Na, Ca, and Fe were also associated with increased antioxidant capacity, and a lower level had adverse consequences. Brown algae, like *Saccharina latissima*, were reported to be used as an alternative to Na content. Similarities in higher concentrations of Na, Ca, and Fe were found. As shown in earlier studies, the increased levels of K, Zn, Cu, and Co were associated with higher antioxidant levels [16]. The variation in agar yield has been reported to differ from species to species, depending on the harvest season.

Two distinct agar formulations were created to ensure agar quality, effectiveness, safety, and stability.  Table 2 shows both the formulation procedures, FA1 is better for *T. conoides* agar formulation. Stability may be influenced by environmental factors such as pH, light, temperature, air, and movement. No change in colour or odour, as well as robust consistency, smooth homogeneity, no microbiological contamination, and sterility, were determined as stability parameters in two different types of FAs. These findings suggest that the two FA gels would be suitable for topical use. There was no evidence pertaining to the phase separation in the two types of FAs during the three-month investigation.

The FT-IR spectrum of FAs extracted from seaweed confirmed the presence of functional groups and bands absorbed in the 4000–500 cm^−1^ ranges are clearly displayed as shown in Figure 2. FAs are confirmed by FT-IR spectra, which showed peaks around 3283.4 cm^−1^ (OH group), 2922.2 cm^−1^ (alkenes), 1829.7 cm^−1^ (C–N stretch), 1496.2 cm^−1^ (alcohols and carboxylic acids), 1038 cm^−1^ (aliphatic amines), and 892 cm^−1^ (aromatics). A considerable absorption band is discovered in 1260 cm^−1^. The existence of S=O bonds in sulphate ester groups explains this. The FT-IR analysis of FAs confirmed the presence of galactopyranose unit and sulphate content indicating the presence of polysaccharides contents which are compared with the standard. All of the FT-IR spectra indicated a broad band ranging from 2900 to 3300 cm^−1^, which is attributed to the O–H stretching vibration from the hydroxyl group of polysaccharides, which corresponded to the hydrophilic property of seaweed [4].

When compared to FA2 (346 kDa), FA1 had a lower molecular weight (205 kDa). The fragmentation spectra of the ions generated from each of the three protonated HexNAcs (m/*z* 150) were compared first. Despite, the fact that both the HexNAcs have the same composition, GalNAc and GalNAc differ from GlcNAc (Figure 3(a) and B) at a single stereocenter [24]. Agaropectin from red algae has a lower molecular weight and sulphate concentration than other agaropectins, with m/*z* = 149 for pentoses, 163 for desoxy-hexoses, and 179 for hexoses. [25].

SEM is used to evaluate the morphology and gel surface of the FAs. SEM images of the plain's exterior surface show it to be flattened, rough, and exceedingly uneven, with a porous structure (Figure 4(a) & 4(b)). The FA1 characteristics' results are present in (Figure 4(a)). It appears to be a smooth, stratified, and ordered flat continuous sheet. Whereas FA2 displayed an irregular, continuous network sheet (Figure 4(b)). According to the findings of Syad et al. [19], the morphological analysis (SEM) extracted from green and brown seaweed has a smooth, flat, and continuous sheet appearance.

The ability of the FA to produce radicals scavenging activities are investigated, as shown in (Table 3). When compared to the antioxidant activities of FA2, FA1 has a significant (*P* < 0.05) increase in antioxidant activities such as DPPH, H_2_O_2_, total antioxidant, and ABTS activities. FA1 has higher sulphate content (41.78%) than FA2(37.25%), which contributes to its high antioxidant activity. Furthermore, when compared to low dose (60 *µ*g/ml) and standard vitamin E, all of the above antioxidant parameters are significantly increased at a high-dose (180 *µ*g/ml) concentration of FA1 and FA2. As a result, significant differences in the in vitro antioxidant, scavenging abilities of phytochemicals isolated from seaweed could be due to differences in the type of extraction and/or the collection zone of the seaweeds [26]. The 180 *μ*l concentration of FA 1 from *T. conoides* showed significant (*P* < 0.05) increase in equal scavenging (82.28 ± 1.09) activity when compared to the concentration of FA2 of 180 *μl* (80.11 ± 0.13). The variations in H_2_O_2_ scavenging percentages in this analysis may be due to differences in extraction techniques or species-specific differences reported in [4]. The ability of the FA to produce total antioxidant activity was investigated, as shown in (Table 3). The 180 *μl* concentration of FA1 from *T. conoides* showed significant (*P* < 0.05) increase equal scavenging (69.65 ± 3.5) activity when compared to the concentration of FA2 of 180 *μl* (64.67 ± 1.41). The capability of the FA to produce ABTS radicals was investigated, as shown in (Table 3). The 180 *μl* concentration of FA1 from *T. conoides* showed significantly (*P* < 0.05) increase equal scavenging (80.66 ± 0.64) activity when compared to the concentration of FA2 of 180 *μl* (72.41 ± 0.35). Considering the absence of phytochemical components, the overall antioxidant activity of *Hypericum olympicum* was found to be very high. This is most likely owing to the presence of other compounds mentioned in the study [20].

The toxicity effects of different concentrations of two FAs with different doses of 0.5 *μg*/ml, 0.25 *μg*/ml, and 0.125 *μg*/ml were evaluated in various aspects. In a low concentration of 0.125 *μ*g/ml, FA1 was less teratogenic when compared with FA2 [22]. It shows the development of embryos for different concentrations of two FAs (control, 0.5 *μ*g/ml, 0.25 *μ*g/ml, and 0.125 *μ*g/ml) at various time periods for different concentrations of two FAs (24 hpf, 48 hpf, 72 hpf, and 96 hpf) (Figure 5(a) and 5(b)). The higher toxicity level resulted in deformities such as yolk sac diffusion, delayed hatching, poor development, and death rate. The lowest concentrations, 0.125 *μ*g/ml and 0.25 *μ*g/ml, showed low pigmentation, tail bending, and body curvature, similarly to the control under constant observation in (Figures 5(a) and 5(b)), and when compared to FA2, the teratogenic activity of the sulphated chitosan, FA1, showed less toxicity in zebrafish larvae [27].

## 4. Conclusion

The agar isolated from *T. conoides* was made into a formulation and FA1 made with more ingredient concentration was found to have higher antioxidant, scavenging activity, and less teratogenicity compared to FA2 made with less ingredient concentration. After clinical trials, the skin permeability of the agar separated may be examined, which could be useful in cosmetic production.

## Figures and Tables

**Figure 1:** Extraction and flow chart of FAs.

**Figure 2:** FT-IR spectrum of FAs.

**Figure 3:** (a, b) GC-MS spectrum of FAs.

**Figure 4:** (a, (b) SEM analysis of FAs.

**Figure 5:** (a, b) Embryotoxicity of FAs.

**Table 1:** Yield and biochemical composition of FAs.

S. no.	Sample	Yield (%)	Sulphate content (%)	Na (%)	K (%)	Mn (%)	Zn (ppm)	Fe (ppm)	Cu (ppm)	Co (ppm)
1	FA 1	84.2	41.78	2.6 ± 0.3	2.7 ± 0.2	20 ± 0.3	51.1 ± 1.0	32.0 ± 1.1	76.01 ± 0.4	3.12 ± 1.3
2	FA 2	80.6	37.25	2.4 ± 0.2	2.5 ± 0.1	18.9 ± 0.2	48.2 ± 1.5	30.3 ± 1.3	73.2 ± 0.5	1.92 ± 1.5

*P* < 0.05, statistical significance.

**Table 2:** Stability of FAs.

S. no.	Parameters/tests	FA1 (25°C ± 2°C) months (0–3)	FA2 (25°C ± 2°C) months (0–3)
1	Colour	Brown colour	Brown colour
2	Odour	No odour change	No odour change
3	pH	6	6.5
4	Consistency	Smooth	Smooth
5	Viscosity (m^2^/s)	0.413	0.61
6	Homogeneity	Good	Good
7	Sterility	No microbial contamination	No microbial contamination
8	Vibrational test	No phase separation	No phase separation
9	Centrifugation test	No phase separation	No phase separation

**Table 3:** *In vitro* antioxidant activities of FAs.

Samples	DPPH scavenging activity (%)	H_2_O_2_ activity (%)	Total antioxidant activity (%)	ABTS activity (%)
FA1 (60 *μ*l)	^*∗*^36.12 ± 0.87	^*∗*^40.18 ± 1.04	^*∗*^20.95 ± 0.83	^*∗*^65.6 ± 0.43
FA1 (120 *μ*l)	69.05 ± 0.9	66.52 ± 2.44	41.31 ± 1.27	66.79 ± 0.16
FA1 (180 *μ*l)	^*∗*^85.14 ± 1.1	^*∗*^82.28 ± 1.09	^*∗*^69.65 ± 3.5	^*∗*^80.66 ± 0.64
FA2 (60 *μ*l)	^*∗*^29.62 ± 0.53	^*∗*^39.40 ± 1.1	^*∗*^20.87 ± 0.09	^*∗*^58.71 ± 1.1
FA2 (120 *μ*l)	65.14 ± 0.9	62.79 ± 0.47	39.17 ± 0.5	64.03 ± 1.67
FA2 (180 *μ*l)	^*∗*^79.7 ± 0.5	^*∗*^80.11 ± 0.13	^*∗*^64.67 ± 1.41	^*∗*^72.41 ± 0.35
Vitamin E (180 *μ*l)	^*∗*^79.86 ± 2.25	^*∗*^77.13 ± 1.91	^*∗*^76.11 ± 3.71	^*∗*^78.50 ± 1.23

∗Statistical significance: *P* < 0.05 (DMRT); ^*∗*^Comparison was made between 180 *µl* of sample and standard.

## Data Availability

All the data generated or analyzed during this study are included in this published article.
